RETRACTED

# Assistive Relief Tool for Early Childhood and Special Psychological Symptom Groups during the Pandemic: Clothing Design Based on the Virtual Contact Principle

**DOI:** 10.1155/2022/9701630

**Published:** 2022-05-20

**Authors:** Yunjuan Liu, Yan Wang, Meiyan Liu

**Affiliations:** ^1^Clothing and Design Faculty, Minjiang University, Fuzhou 350108, China; ^2^Nanchang Key Laboratory of Clothing Digital System Design, Jiangxi Institute of Fashion Technology, Nanchang 330000, China

## Abstract

During the COVID-19 pandemic, some special populations—groups of early childhood and people with autism, among others—faced more profound challenges than the common people. The lack of real physical contact such as embracing greatly affected the effectiveness of development, psychiatric treatment, and other processes for these populations. This study is aimed at developing clothing with appropriate contact pressure based on the contact comfort principle of psychology and providing a type of pressure clothing that can relieve the wearer's tension by simulating hugging, alleviating the lack of physical contact for early childhood education and special education groups during the pandemic. First, the elementary requirements of clothing design are attained using a questionnaire survey and test method. The analysis revealed that clothing should fulfill the four requirements of pressure comfort, fabric softness, wearing and taking off comfort, and visual beauty. Second, we realized the performance requirements in the fabric and accessories, style design, structure design, and functional design. Finally, the product experience is proposed through a fitting, and the reasonable opinions were fed back to the product design to enhance the functionality of clothing. The research shows that clothing can simulate hugging and can ease the loneliness of the wearer. This study can be used as a good tool to assist during the pandemic for early childhood education and special psychological symptom groups, as well as a broader group of people living alone at home, to play an adjunctive treatment and loneliness relief functions.

## 1. Introduction

During the pandemic, the closed and isolated educational environment posed a significant challenge to the effectiveness of online virtual education, especially for the early childhood population and the particular education population (autism and depression).

Unlike adolescents and adults, this group has a greater need for physical contact during the educational process.

Contact comfort, a psychological term, is defined by the American Psychological Association as the positive emotional response of infants and young animals when they come into contact with soft materials; this theory stems from a series of renowned rhesus monkey experiments conducted by American psychologist Harry Harlow [1, 2]. Physical contact like hugging and touching can regulate people's emotions [3, 4]. Specifically, hugging can give people a sense of security and support, can decrease people's sense of fear and loneliness [5, 6], and has several medical functions such as protecting the heart and lowering blood pressure [7]. Contact comfort contributes three interrelated but distinct functions to affective regulation, including social proximity, nursing touch, and intimate contact to regulate emotions [8].

RETRACTED

Some scholars use wearable devices to simulate touch and hug, which are primarily used in online socializing and health. Online socializing is a novel human social organizing and survival mode in the twenty-first century. Based on virtual technology, the communication between people is mostly indirect communication, which lacks physical contact and relies solely on video phone calls and voice chats that affect the maintenance of existing human emotions, especially long-distance lovers, left-behind children, and empty-nest elderly groups [9, 10]. Smart clothing in this field simulates hugging pressure by regulating the tight sense of clothing applied to the wearer's body through electronic information technology to make the wearer feel hugged or touched. For instance, a smart pajama system is available for children called Huggy Pajama [11], which allows parents to control the pajamas worn by their children via the Internet and adjust the air pressure device and heating device in the pajamas, which simulates the pressure and warmth of being hugged, providing children with the feeling of being hugged. Meanwhile, the printing patterns of unique materials used in the clothing can alter the color based on children's emotions, enabling parents to understand children's emotional changes. Similar smart clothes include Sense-Roid [12], HaptiHug [13], and The Hug [14].

In the health domain, mental and psychological issues, such as depression, autism, infantile autism, and mania, have garnered increasing attention. Indeed, some studies have demonstrated that the clinical effect of combined psychotherapy with adjuvant therapy is better than that of conventional drugs, and intelligent clothing with contact comfort is an auxiliary psychotherapy tool [15, 16]. Healthcare personnel suffer from an increased risk of stress, burnout, and depression due to the challenges of the COVID-19 pandemic. Studies show that interactive smart textiles help healthcare workers mitigate their negative feelings [17]. Wearable haptic garments for communicating emotions have great potential in various applications, including supporting social interactions and improving immersive experiences in entertainment [18]. TapTap [19] is a wearable tactile system that uses different driving devices to simulate the leading human touch forms—tapping, pressing, fondling, and touching, and it can be used to train the human tactile sensing system and emotional therapy. Besides, the system can be applied to the pocket scarf, which can be worn on the human body in various ways and can simulate the action of people being hugged and patted around the neck. iFeel_IM! [20] is an implemented system that can considerably enhance the emotionally immersive experience of real-time messaging, reinforcing (intensifying) own feelings and reproducing (simulating) the emotions felt by the partner during online communication through a specially designed system.

RETRACTED

Based on the investigation and analysis of human hugging behavior and hugging contact stress tests, this study is aimed at designing an item of clothing that simulates human contact and hugging to aid in online education for early childhood, people with depression and autism, and other special populations.

## 2. Research Process

First, demand research around two factors: the target audience and clothing. Based on the people's subjective feeling and the function of clothing, as well as considering the clothing comfort, we deduced that the pressure clothing with the function of relieving emotion should have the following four characteristics: provide continuous contact pressure (hugs can relieve stress [21]); have a soft skin touch (skin-friendly to enhance user-friendliness [22]); are easy to put on and take off (functional clothing needs theory [23]); and relieve emotions through color (color relieves stress theory [24]). Second, based on the demand analysis, pressure clothing characteristics were realized through the following four aspects: fabric and accessory design, pattern and color design, structure and process design, and functional design. Finally, we conducted an evaluation study of the pressure clothing prototypes. By trying on two groups of target users, early childhood and depression patients and another group of healthy people, we proposed modifications to the product and fed back to the product design process to improve the design (Figure 1).

## 3. Design Methods

### 3.1. Hugging Behavior Survey

#### 3.1.1. Investigation Contents and Methods

In this study, patients with mild depression and healthy people were selected as research respondents. The questionnaire survey was conducted around personal information, hugging posture, hugging time, and hugging feeling. The key factors to realize the simulation of hugging behavior in pressure clothing design were obtained by investigating and analyzing the information related to hugging behavior.

RETRACTED

The survey covers the needs and preferences of specific users and their concerns. Population classification and questionnaires are used to collect data, which are finally imported into the computer to use quantitative research tools to obtain survey findings. A total of 14 questions were designed, including 2 personal information questions, 5 hugging behavior questions, and 7 hugging psychological feeling questions. We distributed 206 online questionnaires and paper questionnaires and obtained 206 valid questionnaires, with a 100% response rate. Among them, the effective questionnaire respondents included 52 males and 154 females (age: 18–35 years), of whom 42 were patients with mild depression. Of note, the random selection of people enabled observing the difference between different ages and genders in the feeling of hugging. In the questionnaire, the research team set the following content: the self-introduction of the research team and the expression of the purpose of this survey to gain the understanding of the interviewees. In the subject part of the questionnaire, several closed-ended questions were set, and the reverse order of the survey was disrupted according to the relevant content.

#### 3.1.2. Results and Discussion

Taking the survey results and analysis of the question of hugging posture as an example, we presented the analysis process of hugging behavior. The question was designed as “which cuddle position do you find particularly comfortable and enjoyable?” The answer had five options. The results revealed that 46.6% of people thought that face-to-face hugging at the waist was the most comfortable of all (Figure 2). In addition, face-to-face hugging at the waist is called a patting hug (Figure 3), which represents friendship and loyalty. Patting also assists in giving comfort to the other party; however, such an embrace does not have any special intimacy and reveals more about friendship. Thus, hugging psychology is a type of silent communication. Hugging increases our empathy for others and helps the social connection. Perhaps, our results can provide reference information for the distribution of airbags in pressure clothing and that the pressure area should be concentrated in the back of the waist and the front chest.

The overall analysis results of the questionnaire survey revealed that people usually lack hugs in their daily life, but everyone uses a tactile impression to attain environmental information and establish social contact with each other. The most crucial psychological feeling of hugging behavior is warmth, followed by comfort, encouragement, and joy, and few people feel sad after hugging. Hence, hugging can play a vital role in comforting people's tension, and appropriate hugging posture, pressure, and soft touch play a critical role in the comforting effect of hugging and touching.

RETRACTED

### 3.2. Embrace Contact Stress Test

#### 3.2.1. Testing Instruments and Methods

We used the AMI airbag contact pressure tester made in Japan. In the face-to-face hugging posture, the body contact position was chosen as the pressure test point, including three areas of the front chest, with a total of 9 test points, and four areas of the back waist, with a total of 12 test points.

In this study, we selected a total of 53 participants (13 males and 40 females). They hugged each other in pairs to avoid the discomfort caused by hugging a person of the opposite sex. First, the airbag was fixed at 21 test points on a participant, and the participants held each other face-to-face at the waist to find a comfort state and keep it for >30 s. Then, the pressure of 21 test points was read out by a contact pressure testing instrument, and the pressure results of each group were read three times, and the mean value was evaluated.

#### 3.2.2. Results and Analysis

The test demonstrated the distribution of body contact pressure in the face-to-face hugging at the waist (Figure 4).

The experimental results revealed that the pressure exerted on the arm was markedly higher than that on other contact parts. Although the palm often falls on the body of the person being hugged, the arm is the primary force. In the front part of the body, the waist circumference pressure is marginally higher than that of the abdomen and chest; when embracing, the arms are placed around and forcefully increase the contact pressure of the contact area.

Based on the analysis of the test results of hugging contact pressure, the pressure should be >1 kPa in the design of pressure clothing, and the pressure distribution should be adjusted according to body parts.

## 4. Pressure Clothing Design

### 4.1. Airbag Design

Pressure clothing with the function of relieving tension is a type of functional clothing, which can give pressure touch to the human body by inflating the airbag inside the clothing. Together with the test results of the pressure distribution of hugging contact in the previous paper, it is acknowledged that the pressure distribution of the hugged person from large to small is as follows: the back waist of the arm contact part, the back waist of the palm contact, the abdomen, and the chest. Overall, the airbag design should fulfill the following three conditions: (i) the airbags should be equipped at the part of the hugging contact; (ii) the airbags can regulate the contact pressure generated by different parts; and (iii) the airbags can be adjusted per the wearer's body characteristics.

RETRACTED

Figure 5 shows the design of the airbag of this clothing. The airbags include the chest and the back and are connected through webbings. While the front and rear airbags are ventilated separately, the size and thickness of the airbags are different. The skin contact pressure is regulated by the amount of inflation. To adapt to the requirements of different body types and being easy to put on and take off, the length of the webbings is adjusted by the buckles, which regulate the front and rear connection to make the airbags fit the human body better. The airbags are made of white nylon double-bonded TPU (thermoplastic polyurethane) film composite fabric, and the double-layer fabric is segmented into different air storage spaces by the hot-melt method. Notably, different gas storage spaces are not communicated with each other and are connected with the micro air pump by using a gas transmission hose.

### 4.2. Style Design

Figure 6 shows the style. The style features of pressure clothing with relieving emotion function can be summarized as follows: loose blue raglan sleeve sweater; half-open front and middle; and rib edge at the collar, cuff, and hem. The style design primarily considers that the participants should feel comfortable after wearing the clothes and, meanwhile, it can match the airbag well. Thus, choosing blue, the favorite color for nervous people, can calm down their mood. The style should be loose and casual, giving the wearer a relaxed visual sense of ease while being easy to put on and take off. Moreover, the collarless design also decreases the sense of bondage. The half-open design primarily considers the integration of the front chest airbags, and the rib edge has good elasticity, which is convenient to put on and take off without the feeling of tightness.

### 4.3. Fabric Design

The fabric structure is categorized into three layers—outer layer fabric, sandwich adjustable airbags, and lining (Figure 7). The outer layer is prepared of blue elastic knitted fabric, which has good skin touch; its elastic performance can fulfill the requirements of space expansion after the interlayer is inflated. Blue gives people a sense of peace, tranquility, and aloofness, which calms anxiety. The inner layer is made of blue polyester cotton-blended microfiber flannelette, which has the advantages of soft touch and warm feeling. When touching the skin, it can give the wearer a good touch similar to skin contact, which assists in pacifying emotions.

RETRACTED

### 4.4. Functional Evaluation and Teaching Aid Effectiveness Evaluation

#### 4.4.1. Functional Evaluation

The functional evaluation was primarily conducted through the questionnaire survey on the subjective wearing feeling of the participants. The study participants were the same as those in the previous stress testing experiments. The survey contents included the feeling of contact pressure, softness of the fabric, comfort of the style, freedom of putting on and taking off, and presence of the feeling of being hugged.

The feedback is as follows. Regarding clothing acceptance, most people echo that the appearance and color of the clothing are comfortable and beautiful, and it is convenient to put on and take off. It is comfortable to touch by hand. Elastic knitted fabric has good skin touch, and flannelette has a soft touch and warm feeling; they can feel the pressure exerted by the airbags of clothing, feel hugged, and feel relaxed after wearing. However, the pressure clothing feeling differs from person to person; it takes a long time to adjust the pressure, and the pressure contact area is small.

#### 4.4.2. Adjunctive Treatment Effectiveness Evaluation

Early childhood children who were home-isolated for online education during the pandemic and special education students with autism were selected for this research. Feedback was obtained through interviews with parents and psychologists in response to the use of pressure clothing as an aid to online education.

The scenario of the use of pressure clothing is usually accompanied by the psychologists' assessment of the students, instructional activities, etc. The simulated hugging behavior is mostly used to encourage and praise the participants. When virtual hugging behaviors occur in virtual interactions between psychologists and participants, the acceptance rate of participants is high, and also psychologists are more likely to receive good feedback. In contrast, the acceptance rate of the teaching and learning process was generally low if the interaction process was purely online, and there were more instances of nonresponse from the participants.

Secondly, through case studies of incidents of virtual hugging contact behavior occurring during virtual interactions, it can be found that the production of physical contact behavior is mostly not predetermined and has a contextual generative character and that virtual physical contact behavior during participants and psychologists' interactions helps two sides to establish intimate relationships to a certain extent.

Thirdly, most users like to be hugged virtually and are eager for virtual hugs to happen. In fact, all treatment is based on emotional communication. Timely and affectionate hugs from psychologists deliver messages of interaction, making participants feel more secure, eliminating the loneliness of online communication, generating a feeling of being cared for and pampered, and helping learners build confidence. At the same time, to a certain extent, it will not only stimulate participants' desire to communicate emotionally but also satisfy participants' need to socialize as a result of being isolated by the pandemic. In addition, the psychologists give the virtual hug a greater connotation when it is accompanied by an appropriate evaluation of the participants.

RETRACTED

## 5. Summary and the Way Forward

The virtual contact pressure clothing is an effective attempt to complement the special online education for isolation during a pandemic. The design and development of pressure clothing that can relieve the wearer's emotion is based on the contact comfort principle of physiological psychology. Contact pressure and contact softness are the two factors that play a role in skin contact comfort. By adding airbags in the garment interlayer and soft touch of fabric, the human body feeling of hugging was simulated in this study, and the design was executed from the aspects of clothing comfort and visual beauty. This garment principally realizes that the wearer feels embraced, making the wearer feel comfortable and secure to some extent. Both the functional evaluation and the actual teaching effectiveness evaluation studies have been positively evaluated by users.

The analysis of the feedback results of the fitting experiment deduced that there exist some aspects to be enhanced in this functional clothing design. First, the pressure-increasing speed of airbags inside the garment is slow. Second, the garment can only simulate one touch and hug posture. Third, the clothing lacks the parts that can provide head and neck support, which decreases the comfort. To solve these problems, the intelligent control module should be added in the subsequent design to materialize the objective of rapid pressure increment and flexible pressure control. Meanwhile, in the style design, the airbag distribution position should be enhanced, the multichannel pressure should be applied to realize the purpose of simulating all types of hugging posture, and the neck support component should be added to make the wearer's head feel dependent on the shoulder of the other party.

## Figures and Tables

**Figure 1:** Research process.

**Figure 2:** Analysis results of “hug posture preference.”

**Figure 3:** Diagram of face-to-face hugging at the waist.

RETRACTED

**Figure 4:** Distribution of body contact pressure in the face-to-face hugging at the waist.

**Figure 5:** Schematic diagram of airbag design.

**Figure 6:** Style diagram.

**Figure 7:** Fabric layer distribution diagram.

## Data Availability

The data used to support the findings of this study are available from the corresponding author upon request.
